# Cardiac External Counterpulsation Attenuates Myocardial Injury by Regulating NRF2-mediated Ferroptosisin and Oxidative stress Injury

This article has been retracted.

**DOI:** 10.1155/2022/6477778

**Published:** 2022-10-10

**Authors:** ShiXiang Wang, Bin Wang, Guofeng Guo, Youquan Chen

**Affiliations:** ^1^Department of Cardiovascular Medicine, The Third Affiliated Hospital of Guangzhou Medical University, Guangzhou 510150, Guangdong, China; ^2^Department of Radiology, Heze Hospital of Traditional Chinese Medicine, Heze 274400, Shandong, China

## Abstract

**Objectives:**

To explore the role of the external counterpulsation (ECP) myocardial injury by controlling NRF2-mediated ferroptosis and oxidative stress damage in acute myocardial infarction.

**Methods:**

Twenty acute myocardial infarction (AMI) participants hospitalized from January 2021 to January 2022 were enrolled. In addition, 20 healthy individuals who had a physical examination at our hospital served as normal controls. Before the AMI patients were given ECP therapy, the blood samples were collected and echocardiography was performed as the data of AMI cohort. Then, the blood samples were collected and echocardiography was performed following the ECP therapy as the data of AMI + ECP cohort. The heart function was assessed by echocardiography test.

**Results:**

Our findings demonstrated that ECP could reduce heart damage in patients with AMI. In the current study, we found that ECP could reduce heart damage in patients with AMI through increasing the LV-EF% and enhancing LVEDV and LVESV, and the difference was statistically significant (*P* < 0.05). ECP could reduce the levels of oxidative stress and ferroptosis markers in blood samples of AMI patients, which was through the upregulation of NRF2 and HO-1 expression, and the difference was statistically significant (*P* < 0.05). Taken together, all data implied that ECP was able to attenuate myocardial injury by regulating NRF2-mediated ferroptosis and oxidative stress in AMI patients, and the difference was statistically significant (*P* < 0.05).

**Conclusion:**

Our findings in this research are that cardiac ECP is able to attenuate myocardial injury by regulating NRF2-mediated ferroptosis and oxidative stress injury in AMI patients. This certainly gives the possibility of a clinically effective treatment for AMI patients, although further clinical trials need to be validated.

## 1. Introduce

Acute myocardial infarction (AMI) is a leading contributor to fatalities and morbidities throughout the world [1]. Each year approximately 10% of people admitted to the emergency department with chest pain are given a diagnosis of cardiac arrest [2–4]. Presently, no therapeutic options are available to prevention of ischemic reperfusion injuries (IRI) in the heart, which leads to the need for an in-depth investigation of the pathophysiology. Many works have demonstrated that oxidative stress is the predominant reason for IRI, which can upregulate the generation of reactive oxygen species (ROS), driving the pathogenesis of IRI [5, 6]. Moreover, an additional essential source is the imbalance of iron homeostasis, which will result in an elevated level of free iron in the cardiomyocytes. This metal ion will be elevated by the release of hydroxyl radicals (-OH) through the Fenton reaction. Eventually, these activators accelerate cellular damage by attacking biomolecules, such as lipids and proteins, and initiating various cell death pathways [7]. AMI is a disorder that can be co-occurring with ischemic cardiopathy and is manifested when atherosclerotic plaques rupture and a growing blood clot entirely or partially occludes a crown artery, limiting circulation to the heart.

NRF2 is a stress-induced transcription factor in which protein levels are maintained at essentially a low level by three distinct E3-ubiquitin ligase enzymatic complexes [8]. External counterpulsation (ECP) therapy is a noninvasive assisted cardiovascular apparatus that is approved by the U.S. Food and Drug Administration for refractory angina pectoris. Remarkably, many proteins and enzymes responsible for the prevention of lipid peroxidation, and the resulting initiation of iron toxicity, are the target genes of NRF2. NRF2/HO-1 is a property found in almost 100% of human cells. It is triggered, relocated to the nucleus, and bound to DNA via antioxidant-response elements (AREs). As a modulator of the antioxidative response system, it upregulates the expression of HO-1 to minimize oxidative stress [9]. Previous investigations have proven the clinical applications of NRF2/HO-1 in pediatric cardiovascular disorders [9].

As a result of genetic mutations, endogenous stress-induced modifications, competitive conjugation of other interacting partners, or exogenous pharmacological inhibition, NRF2 can then translocate to the nucleus and initiate transcription of genes containing antioxidant-response elements (ARE) [10]. It is insufflated in the inferior extremities to raise the diastolic pressure in the aorta, thus augmenting the coronary perfusion. The cuff is deflated under systole to decrease vessel compression and heart backload. The increased hemodynamics and velocity of flow generate a shearing strain on the endothelium, resulting in improved functionality of the endothelium. In individuals with coronary artery disease (CAD), ECP is capability of triggering the release of nitric oxide, a vasodilator, and diminishing those vasoconstrictors [11, 12]. Thus, the modulation of these pathways by a shear force in the endothelium may attenuate the progression of cardiovascular disease. However, the influence of ECP in ferroptosis and oxidative stress has not remained unclear to the mitigation of myocardial injury via NRF2/HO-1. This study was to explore the role of ECP in myocardial injury by controlling NRF2-mediated ferroptosis and oxidative stress damage in acute myocardial infarction.

## 2. The Information of Patients and Methods

### 2.1. General Information of Participants

Twenty AMI participants hospitalized from January 2021 to January 2022 were enrolled in current research. In addition, 20 healthy individuals who had a physical examination at our hospital served as normal controls. There exhibited no remarkable difference in general data between AMI patients and normal cases. Before the AMI patients were given ECP therapy, the blood samples were collected and echocardiography was performed as the data of AMI cohort. Then, the blood samples were collected and echocardiography was performed following the ECP therapy as the data of AMI + ECP cohort. Our study has been approved by the hospital's ethics committee. All patients have signed an informed consent form.

### 2.2. Echocardiography

Left ventricular end-diastolic volume (LVEDV, ml), left ventricular end-systolic volume (LVESV, ml), and left ventricular ejection fraction (LV-EF, %) were measured by echocardiography. The date among normal controls, AMI cohort, and AMI + ECP cohort were taken as comparisons to assess the cardiac functions.

### 2.3. ELISA Assay

All plasma was obtained from the blood samples. The evaluation of oxidative stress was verified via measurement of superoxide dismutase (SOD), glutathione peroxidase (GPx), catalase and reduced glutathione (GSH), and malondialdehyde (MDA) by using an ELISA kit (Lifespan Biosciences, USA). All experimental practices were performed according to the manufacturer's protocol. The experiment was repeated three times.

### 2.4. RT-qPCR Assay

For this test, *β*-actin was utilized as an internal reference gene and the mRNA expressed each gene was determined using the 2^−ΔΔct^ relative quantification approach and standardized to the expressed relative to the control group. At least a minimum of triple testing was replicated. Complete RNA was derived from the blood of both healthy volunteers and patients pre- and post-ECP treatment using TRIzol reagent (Takara, Japan) and reversely transcribed into cDNA in a cDNA synthesis kit (Takara). Quantitative PCR was undertaken on the Ultra SYBR One-StepRT-qPCR Kit (CWBIO, China) and gene-specific primers. The quantity of RNA was counted using the comparative threshold cycling method. All primers were customized by GenScript, Inc. The primers of ACSL4, TFR1, GPX4, NRF2, and HO-1 are displayed in Table 1.

### 2.5. Iron Content Measured by ELISA

For quantitative determination of iron Fe^3+^ and/or Fe^2+^, the evaluation of iron metabolism was conducted using QuantiChrom™ Iron Assay Kit (Bio Assay Systems, US) by following the manufacturer's instructions. The blood samples were collected, homogenized in 5x volume of iron assay buffer on ice, and centrifuged (13,000 × *g*, 10 min) at 4°C. The supernatant was collected, and 5 *μ*l of iron reducer was added to each sample and incubated for 30 min at 37°C. Next, 100 *μ*l of iron probe was added to each sample and incubated for 60 min at 37°C away from light. The intensity of the color was measured at 590 nm. A minimum of triple testing was replicated at least.

### 2.6. Statistical Analysis

IBMSPSS24.0 software was applied for statistical analysis. The measurement data were expressed by mean ± standard deviation. The counting data were expressed by frequency or rate. *T*-test was used when measurement data obey normal distribution, and rank sum test was used when it did not obey normal distribution. *χ*2 test was used to compare the classified counting data. Repeated measurement data were analyzed by repeated measurement analysis of variance. Main effect test results were used when there was no interaction, and simple effect analysis was carried out when there was an interaction. *P* < 0.05 indicated that the difference between groups is statistically significant.

## 3. Results

### 3.1. ECP Could Reduce Cardiac Damages in Patients with AMI Compared with Controls

Following the ECP treatment to the AMI patients, LV-EF% of AMI + ECP cohort was increased remarkably than pre-ECP therapy (Figure 1(a)), and the difference was statistically significant (*P* < 0.05). However, LV-EF% of AMI + ECP cohort still showed lower than the normal controls, and the difference was statistically significant (*P* < 0.05). LVEDV and LVESV were upregulated after ECP therapy, which were considerably relieved before ECP therapy, and the difference was statistically significant (*P* < 0.05). In addition, there was no obvious distinction between normal controls and patients of AMI + ECP cohort (See Figures 1(b) and 1(c)). These data released that ECP could reduce heart damage in patients with AMI.

### 3.2. ECP Could Reduce the Levels of Oxidative-Stress Markers in Blood Samples of AMI Patients

The oxidative-stress biomarkers were assessed among controls, AMI, and AMI + ECP cohorts. The current data suggested that MDA and SOD levels of AMI cases were considerably higher than healthy control participants, and the difference was statistically significant (*P* < 0.05). However, MDA and SOD values were downregulated remarkably after ECP treatment, and the difference was statistically significant (*P* < 0.05). On the other hand, GSH and GPx were obviously raised than healthy cases when the patients were suffering from AMI, and the difference was statistically significant (*P* < 0.05). Following the ECP therapy, GSH and GPx levels of AMI + ECP cohort were improved obviously than pre-ECP treatment, and the difference was statistically significant (*P* < 0.05). Taken together, these results imply that ECP could reduce the levels of oxidative-stress markers in blood samples of AMI patients (Figure 2).

### 3.3. ECP Could Downregulate Levels of Ferroptosis in Blood Samples of AMI Patients

The level of plasma iron content was upregulated considerably when the cases were suffering from AMI. After ECP treatment, the plasma iron content was reduced obviously than AMI patients, and the difference was statistically significant (*P* < 0.05). In addition, the levels of ACSL4 and TFR1 were strongly expressed, while the GPX4 expression decreased in AMI patients than the normal healthy group, and the difference was statistically significant (*P* < 0.05). In AMI + ECP cohort, the expressed ACSL4 and TFR1 mRNA was suppressed remarkably, at the meanwhile, the GPX4 mRNA level was weakened greatly, and the difference was statistically significant (*P* < 0.05). All the data suggested that ECP therapy could downregulate markers of ferroptosis in blood samples of AMI patients (Figure 3).

### 3.4. ECP Could Activate the NRF2/HO-1 Pathway in Blood Samples of AMI Patients

Before the therapy of ECP to AMI patients, the lower expressions of NRF2 and HO-1 levels were exhibited in AMI cases than that in normal controls, and the difference was statistically significant (*P* < 0.05). However, the levels of NRF2 and HO-1 were evaluated after the patients accepted the ECP therapy (See Figure 4).

## 4. Discussion

In the current study, we found that ECP could reduce heart damage in patients with AMI through increasing the LV-EF% and enhancing LVEDV and LVESV. ECP could reduce the levels of oxidative stress and ferroptosis markers in blood samples of AMI patients, which was through the upregulation of NRF2 and HO-1 expression. Taken together, all data implied that ECP was able to attenuate myocardial injury by regulating NRF2-mediated ferroptosis and oxidative stress in AMI patients. This study was to explore the role of the external counterpulsation (ECP) myocardial injury by controlling NRF2-mediated ferroptosis and oxidative stress damage in acute myocardial infarction.

The management of myocardial infarction has greatly advanced in the previous four decades [3, 13]. Consequently, it has grown more widespread for patients to have survived the acute event. Medically indicated remedies to limit infarct size are vital, as massive infarcts can contribute to cardiogenic shock, fatal arrhythmias, or acute heart failure [14–16]. During reperfusion, cardiomyocytes are submitted to further oxidative stress, a mandatory process for myocardial resuscitation [17, 18]. This impairment, thought to be ischemia-reperfusion, contributes to a submerged wave of cell death and an inflammatory reaction. ROS generated during and after ischemia and reperfusion are thought to be the main cause of cell death.

Medications that decrease cell mortality are predicted to lessen infarct size, preventing adverse events and having tremendous clinical implications. The initial ischemia at the cytosolic level can result in an elevation of reactive oxygen species (ROS). The free radicals are generated as by-products of regular cell metabolism, and the elevated levels of ROS may result from enhanced productivity or diminished damage to such formed free radicals by enzymatic and nonenzymatic antioxidants [19]. Alteration in the enzymatic levels of these antioxidants can seriously influence the sensitization of diverse organs to oxidative stress and is consequently involved in myocardial damage [20]. Current results demonstrated that MDA and SOD levels of AMI cases were considerably higher than healthy control participants. However, MDA and SOD values were downregulated remarkably after ECP treatment. On the other hand, GSH and GPx were obviously raised than healthy cases when the patients were suffering from AMI. Following the ECP therapy, GSH and GPx levels of AMI + ECP cohort were improved obviously than pre-ECP treatment. MDA and SOD were assessed as oxidative stress markers. The generation of oxidative free radicals and the magnitude of tissue impairment can be reflected indirectly by the measurement of lipid peroxidation and MDA [21]. SOD is an enzyme that cleaves the superoxide anion radical O_2_- and has a major part in oxidation and antioxidation homeostasis in the body [22]. The alteration of serum MDA and SOD levels were in accordance with the apoptotic activity, while GSH and GPx activities exhibited the contrary pattern, indicating that the underlying therapeutic principle of AMI may be associated with antiapoptotic effect and oxidative stress [23]. Ferroptosis is primarily characterized by mitochondrial atrophy, in which the density of bilayer membranes improves and lipid peroxidation is accumulated. Myocardial ischemia-reperfusion injury (MIRI) is an unavoidable risk event for acute myocardial infarction. This part of the results implies that ECP can improve the function of injured myocardium, possibly through oxidative stress.

Ferroptosis is a newfound regulatory state form of cytosolic death depending on iron and ROS [24, 25]. It directly or indirectly influences GPX4 by induction of smaller molecules, which causes an overaccumulation of ROS in membrane-lipids due to redox inequality and damages the integrity of cytosolic membranes [26, 27]. Ferroptosis is closely associated with MIRI [28]. After ECP treatment, the plasma iron content was reduced obviously than AMI patients. In addition, the levels of ACSL4 and TFR1 were strongly expressed, while the GPX4 expression decreased in AMI patients than the normal healthy group. In AMI + ECP cohort, the expressed ACSL4 and TFR1 mRNA was suppressed remarkably, at the meanwhile, the GPX4 mRNA level was weakened greatly. All the data suggested that ECP therapy could downregulate markers of ferroptosis in blood samples of AMI patients. ACSL4 and GPX4 are considered to be central factors participating in lipid peroxidation [29]. ACSL4 is a representative of the long-chain series of acyl-CoA synthetases that initiate long-chain fatty acids to produce cytosolic lipids, while GPX4 is thought to be the major enzyme that suppresses ferroptosis by transforming lipid hydroperoxide into nontoxic lipid alcohols [30]. Former investigations have indicated that ACSL4 is essential for the triggering of iron atrophy and that suppression of ACSL4 inhibits the occurrence of iron atrophy [30]. The translational element NRF2, which is encoded by the NFE2L2 gene, is most well-known for controlling the performance of antioxidant and detoxifying genes. Gene-knockout approaches have proven its general cytoprotective properties. It is featured by its reliance on iron and the accumulated lipid peroxides. TfR1 and iron phagosome have been determined to be essential modulators of iron accretion. TfR1 are membrane-based proteins that translocate iron from the extracellular surroundings into the cell and facilitate the building of the cellular iron pool required for ferroptosis [31].

NRF2 has been the subject of intensive research in cancer biology since its discovery in 1994, and the comprehension of the effect of NRF2 in cardiovascular disorders is just emerging [32]. Our current results displayed that before the therapy of ECP to AMI patients, the lower expressions of NRF2 and HO-1 levels were exhibited in AMI cases than that in normal controls. However, the levels of NRF2 and HO-1 were evaluated after the patients accepted the ECP therapy. It is proven that ECP could activate the NRF2 pathway in blood samples of AMI patients. There are some limitations in this study. First, the sample size of this study is not large and it is a single-center study, so bias is inevitable. In future research, we will carry out multicenter, large-sample prospective studies, or more valuable conclusions can be drawn.

## 5. Conclusion

In conclusion, our findings in this research are that cardiac ECP is able to attenuate myocardial injury by regulating NRF2-mediated ferroptosis and oxidative stress injury in AMI patients. This certainly gives the possibility of a clinically effective treatment for AMI patients, although further clinical trials need to be validated.

## Figures and Tables

**Figure 1:** ECP could reduce heart damage in patients with AMI. LVEDV, LVESV, and LV-EF % were measured by echocardiography. ^*∗∗∗*^*P* < 0.001 (control vs. AMI); ^&^*P* < 0.05, ^&&^*P* < 0.01(AMI vs. AMI + ECP).

**Figure 2:** ECP could reduce oxidative-stress markers in blood samples of AMI patients. MDA (a), GSH (b), GPx (c), and SOD (d) were measured by ELISA. ^*∗∗∗*^*P* < 0.001 (control vs. AMI); ^&&&^*P* < 0.001 (AMI vs. AMI + ECP).

**Figure 3:** ECP could downregulate markers of ferroptosis in blood samples of AMI patients. Iron content (a) was measured by ELISA. The mRNA expressions of ACSL4 (b), TFR1 (c), and GPX4 (d) were measured by RT-qPCR. ^*∗∗∗*^*P* < 0.001 (control vs. AMI); ^&&^*P* < 0.01 ^&&&^*P* < 0.001(AMI vs. AMI + ECP).

**Figure 4:** ECP could activate the NRF2 pathway in blood samples of AMI patients. The mRNA expressions of NRF2 (a) and HO-1(b) were measured by RT-qPCR. ^*∗*^*P* < 0.05, and ^*∗∗∗*^*P* < 0.001 (control vs. AMI); ^&&^*P* < 0.01 ^&&&^*P* < 0.001(AMI vs. AMI + ECP).

**Table 1:** Primer sequences used for qPCR.

Gene		Sequence (5′ to 3′)
*β*-actin	F	GCACCCAGCACGATGAAAAT
	R	GACAATGGAGGGTCCGGATT
ACSL4	F	ATATTCGTCACCACTCACA
	R	AACCTTGCTCATAACATTCTT
TFR1	F	AGAATGGCTGGAGGGGTACT
	R	TTCTCTCCAGCAGCGCATAC
GPX4	F	CAGGAGCCAGGAAGTAAT
	R	CAGCCGTTCTTATCAATGAG
NRF2	F	GCCCACATTCCCAAACAAGAT
	R	CCAGAGAGCTATTGAGGGACTG
HO-1	F	GCAGAGGGTGATAGAAGAGG
	R	AAGGAAGCCAGCCAAGAG

## Data Availability

The datasets used and analyzed during the current study are available from the corresponding author upon reasonable request.
